# Intermittent Hypoxia and Atherosclerosis: From Molecular Mechanisms to the Therapeutic Treatment

**DOI:** 10.1155/2022/1438470

**Published:** 2022-08-03

**Authors:** Binyu Luo, Yiwen Li, Mengmeng Zhu, Jing Cui, Yanfei Liu, Yue Liu

**Affiliations:** ^1^National Clinical Research Center for Chinese Medicine Cardiology, Xiyuan Hospital, Chinese Academy of Chinese Medical Sciences, Beijing 100091, China; ^2^The Second Department of Gerontology, Xiyuan Hospital, China Academy of Chinese Medical Sciences, Beijing 100091, China

## Abstract

Intermittent hypoxia (IH) has a dual nature. On the one hand, chronic IH (CIH) is an important pathologic feature of obstructive sleep apnea (OSA) syndrome (OSAS), and many studies have confirmed that OSA-related CIH (OSA-CIH) has atherogenic effects involving complex and interacting mechanisms. Limited preventive and treatment methods are currently available for this condition. On the other hand, non-OSA-related IH has beneficial or detrimental effects on the body, depending on the degree, duration, and cyclic cycle of hypoxia. It includes two main states: intermittent hypoxia in a simulated plateau environment and intermittent hypoxia in a normobaric environment. In this paper, we compare the two types of IH and summarizes the pathologic mechanisms and research advances in the treatment of OSA-CIH-induced atherosclerosis (AS), to provide evidence for the systematic prevention and treatment of OSAS-related AS.

## 1. Introduction

Intermittent hypoxia (IH) refers to a state of repeated hypoxia–reoxygenation alternating with periods of normoxia. In particular, chronic IH (CIH) mostly occurs in patients with obstructive sleep apnea (OSA) syndrome (OSAS) and is an important pathologic feature of OSAS [1–3], causing damage to multiple systems such as the cardiovascular, nervous, respiratory, circulatory, and endocrine systems.

The disease background of CIH is homogeneous and is mostly seen in patients with OSA. Compared with OSA-CIH, the research background of other types of IH is more complex, and there is no relatively unified and accepted research model, so they are uniformly classified as non-OSA-IH in this paper. Some non-OSA-IH models can have positive effects such as improving the hypoxia tolerance of the body and alleviating cardiac ischemia–reperfusion injury [4], suggesting that different IH patterns can mediate different biological effects.

Patients with OSAS who are exposed to CIH are at an increased risk of developing several major risk factors for atherosclerosis (AS), including obesity, hyperglycemia, hypertension, and dyslipidemia [5–7]. The association between intermittent hypoxia and atherosclerosis has been studied more frequently, but relatively few studies have been conducted on persistent hypoxia and atherosclerosis. The study [8] found that hypoxia induced proliferation of smooth muscle cells and plaque formation in the aorta of ApoE^−/−^ mice after 3 weeks of feeding in a gas chamber with hypoxia (10.0 ± 0.5% O_2_), but not in normoxia. Smooth muscle cell proliferation and plaque formation were found to be induced by hypoxia, but not by normoxia, along with an increase in plasma LDL cholesterol, NADPH-dependent vascular superoxide (O^2-^), and activation of matrix metalloproteinase 9. Thus, this study not only confirms that chronic sustained hypoxia accelerates the development of atherosclerosis, but also suggests possible mechanisms, such as abnormal lipid metabolism and reactive oxygen species production. We focus on the interrelationship between OSA-IH and AS. The study of sustained hypoxia and AS will be discussed specifically in future studies.

This article will focus on the bidirectional clinical impact of IH, the pathologic mechanisms by which OSA-CIH causes AS, and the current research advances in treatment methods, with the aim of providing a reference for the prevention and treatment of AS secondary to OSAS.

## 2. Dual Nature of IH

There are several different models of IH, capable of producing positive or negative effects on the organism, i.e., the two-sided nature of IH. Most cases of OSA-related IH are chronic (i.e., OSA-CIH), which can induce the onset of AS and hence produce various pathologic outcomes. Non-OSA-IH can exert different effects on the body depending on its intensity; that is, low-intensity IH can have several protective effects, whereas high-intensity IH mostly leads to adverse consequences, which suggests that the physiologic effects of IH are correlated with its intensity [9]. In the non-OSA-IH paradigm, central sleep apnea (CSA) as a sleep disorder is mostly a chronic process with a complex classification and different effects on the organism. Our discussion of non-OSA-IH is dominated by patterns that bring positive effects to the organism (see Table 1 and Figure 1).

### 2.1. OSA-CIH

OSA is mainly characterized by upper airway obstruction during sleep and discontinuous nighttime sleep, leading to repeated hypoxia-reoxygenation cycles that last from weeks to years, resulting in CIH. Upper airway narrowing is an important structural basis for this. The cross-sectional area of the pharyngeal airway is significantly reduced in OSA patients compared to non-OSA patients [24]. OSA-CIH can promote oxidative stress by increasing ROS expression, inflammation by increasing NF-*κ*B activity, and blood pressure elevation and inflammatory response by increasing carotid body-mediated sympathetic activity [25], which leads to a variety of cardiovascular and cerebrovascular diseases occurrence and development. Patients with OSAS tend to have a chronic course of disease. Their hypoxic state usually manifests as CIH (characterized by a long duration of severe hypoxia with a high frequency of episodes and short cycles), which can result in a wide range of adverse consequences. For example, OSA-CIH can significantly increase the morbidity and mortality of various diseases and is an independent risk factor for cardiovascular diseases [26]. OSA was found to be significantly correlated with the incidence and severity of hypertension [27]. A cross-sectional study covering 2677 adults showed that the number of patients with hypertension increased linearly with the severity of OSA and that each increase in sleep apnea was associated with a 1% increase in the odds of developing hypertension [28]. A first retrospective study describing comorbidities in Hungarian and Romanian OSA patients showed that various diseases such as cardiovascular diseases (e.g., hypertension and arrhythmias), diabetes, and asthma were strongly associated with OSA severity in the whole study population and that OSA-CIH played an important role in it [29]. Khamsai et al. found that patients with OSA combined with hypertension were much more likely to develop hypertensive crisis than the general population [30], greatly increasing the risk of various cardiovascular and cerebrovascular diseases. It was also noted that carotid artery intima-media thickness and AS-related inflammatory markers were significantly increased in hypertensive patients with combined OSA, confirming the damage to the vascular endothelium caused by this pathological phenomenon [31]. In addition, the risk of atrial fibrillation is significantly increased by OSA-CIH and exponentially increased by the presence of both OSAS and heart failure [32–38]. OSA-CIH can also facilitate the development of coronary heart disease [39], heart failure [40], and aortic dissection [41]. Among them, OSA was significantly associated with the incidence of aortic coarctation. A meta-analysis noted an increased risk of up to 433% between moderate-to-severe OSA and aortic coarctation, but the incidence of aortic coarctation in patients with OSA has not been derived due to the relatively short follow-up period of the study [42]. In terms of metabolic diseases, a meta-analysis [43] revealed that moderate-to-severe OSA was associated with an increased incidence of type 2 diabetes mellitus. This may be because OSA-CIH can cause glucose metabolic disorders by increasing oxidative stress (OS) and inflammation and can directly affect the pancreatic *β*-cells, liver, and other organs and tissues, thereby influencing glucose homeostasis [44]. Furthermore, this hypoxic pattern can lead to liver fibrosis, inflammation, and liver damage by inducing inflammatory mediators such as nuclear factors, resulting in hepatic dyslipidemia that can further develop into nonalcoholic fatty liver disease [45]. Therefore, OSA-CIH plays an important role in promoting the development of many AS-related diseases.

### 2.2. Non-OSA-IH

The effects of non-OSA-IH on the organism are closely related to the duration, frequency, and degree of hypoxia: short, low-frequency, and mild hypoxia usually has a protective effect on the organism, while the opposite causes damage to the organism [9].

The current research on non-OSA-IH mainly includes three types of intermittent low-pressure hypoxia, intermittent normobaric hypoxia, and CSA related IH, which can have different effects on the organism depending on the duration, frequency, and cyclic cycle of hypoxia. Each of them will be discussed in the following section.

Many studies have found that residents of high altitude areas have a relatively low incidence of heart attacks and coronary heart disease mortality [46]. Therefore, many scholars have found that such intermittent hypoxia has various protective effects on the organism after intermittent low-pressure hypoxia training in a low-pressure chamber (4-8 hours per day, with the rest of the day at atmospheric pressure) simulating a high-altitude environment. For example, when expedition members underwent IH training in a hypobaric chamber at a simulated altitude of 4000–5500 m, their time spent exercising significantly increased, and their erythrocyte, reticulocyte, and platelet counts were found to be elevated [19]. These findings suggest that this type of IH can enhance the oxygen-carrying capacity and tolerance to ischemia and hypoxia of tissues, thus improving exercise endurance. Left ventricular function was assessed in isolated hearts of rats treated with similar chronic intermittent low-pressure hypoxia (CIHH, at an altitude of 3000 m, CIH environment). It was found that after treatment of isolated hearts with ischemia/reperfusion injury, the recovery of cardiac function was significantly enhanced in CIHH rats compared with controls, and they had higher superoxide dismutase levels and total antioxidant capacity. These protective effects were counteracted by the addition of an ATP-sensitive potassium (KATP) channel inhibitor, a mitochondrial KATP inhibitor, and a mitochondrial permeability transition pore opener. This study not only demonstrated the protective effect of CIH, but also verified for the first time that this effect was associated with KATP channels [14] In addition to the cardiac benefits, intermittent low-pressure hypoxic training has been shown to contribute to weight loss and glycemic control in prediabetic obese patients and is expected to help restore normal fasting glucose in prediabetic patients [47].

Central sleep apnea occurs when the drive to breathe by the medullary respiratory center is temporarily stopped resulting in the disappearance of both oral and nasal airflow and thoracic and abdominal movements. Its classification is complex and includes primary central sleep apnea, central sleep apnea due to Cheyne-Stokes breathing pattern, and central sleep apnea due to high altitude periodic breathing. Unlike the intermittent hypoxia that simulates a high altitude environment above, travelers to high altitudes are in a continuous hypoxic state for a specific period of time and usually experience central sleep apnea, which manifests as restless sleep and nonresolving sleep upon awakening. Hyperventilation occurs after exposure to hypoxia and increases with time, usually after about 10 minutes of hypoxia in the form of gradual strengthening-decreasing respiration, with a gradual increase in respiratory amplitude, resulting in a gradual decrease in PaCO2 and an apnea, followed by an increase in inspiration, and so on and so forth, showing periodic breathing. The main mechanism is hypoxemia. Chronic respiratory stimulants and CO2 inhalation can reduce or even eliminate this periodic respiration [48].

Multiple factors can contribute to the development of CSA and often coexist with OSA, making the classification complex. CSA is associated with a variety of diseases, such as heart failure, renal failure, and stroke. Similar to OSA, CSA is also associated with intermittent hypoxia, but due to the complexity of the respiratory pattern and the diversity of classification of CSA, there are few animal studies on CSA-IH, and a relatively perfect animal model cannot be summarized for reference. In contrast, the animal model of OSA is relatively simple to construct, so most of the current animal studies on IH use OSA as the research background, and Table 1 is also compiled through these literatures.

In addition to the low-pressure environment similar to the plateau environment, IH at atmospheric pressure has also been shown to have positive effects [49, 50]. For example, IH can improve mitochondrial efficiency and enhance tissue perfusion by activating hypoxia-inducible factor 1*α* (HIF-1*α*), which enhances muscle oxygen homeostasis [51–53]. In addition, under IH conditions, blood pressure in hypertensive patients is significantly reduced or even normalized [54, 55]. A study conducted in patients with stage I hypertension demonstrated for the first time that IH conditioning can lower blood pressure by affecting nitric oxide (NO) synthesis. Hence, IH conditioning can be a nonpharmacologic treatment option for patients with stage I hypertension [55]. Furthermore, IH preconditioning in rats [50] and dogs [56] led to a reduction in infarct size in both animal models, as well as to a lower incidence of ventricular arrhythmias in dogs. This protective effect may be achieved through increased NO production or adrenergic receptor activation [56].

In addition, non-OSA-IH can improve neurocognitive function [57], enhance innate immunity [58], and induce endogenous cardioprotection through oxidative stress [59]. Hence, it is expected to provide new ideas and methods for the treatment of many diseases.

## 3. Pathophysiologic Mechanisms Underlying OSA-CIH-Induced AS

### 3.1. Inflammation

Because inflammation plays a crucial role in AS development, AS is considered a chronic inflammatory disease [60, 61]. Studies have shown that CIH can induce AS through the activation of inflammatory [62] pathways, including HIF, nuclear factor kappa-B (NF-*κ*B), and Toll-like receptor 4 (TLR4).

HIF belongs to the family of transcriptional activators. HIF-1, the first member of its family to be identified, consists of oxygen-sensitive HIF-1*α* and constitutively expressed HIF-1*β*, which are present in all mammalian cells and are able to respond sensitively to hypoxic environments [63, 64]. Animal studies have found that CIH significantly upregulates HIF-1*α* levels in vivo [65]. HIF-1*α* has been clearly demonstrated to be associated with atherosclerosis: it promotes macrophage activation and conversion into proinflammatory cells, releasing IL, TNF, and other cytokines, which have an impact on plaque formation and stability [66]. In vivo studies in LDL^−/−^ mice have found that HIF-1*α* deficiency in bone marrow cells substantially reduces atherosclerosis by a mechanism associated with HIF-1*α* affecting its inflammatory properties [67]. In addition, HIF-1*α* can also promote the formation and development of atherosclerosis by affecting glucose metabolism and apoptosis of macrophages, migration and proliferation of vascular smooth muscle cells, and permeability of endothelial cells [68].

The NF-*κ*B pathway is one of the major inflammatory pathways. One study [69] found that CIH exposure not only increased NF-*κ*B binding activity in a time-dependent manner across multiple organs and tissues in mice but also increased the expression of inducible NO synthase, an NF-*κ*B-dependent gene product. Furthermore, patients with OSAS showed significantly increased monocyte NF-*κ*B activity compared with controls, which significantly decreased when their CIH was corrected. These findings suggest that CIH is an important pathologic mechanism leading to NF-*κ*B activation in patients with OSAS. In an experimental study [70], CIH + a high-cholesterol diet (HCD) induced AS development, whereas knockdown of the NF-*κ*B P50 subunit eliminated the AS lesions induced by CIH + HCD by significantly inhibiting three major atherogenic mechanisms: vascular inflammation, hypercholesterolemia, and macrophage foam cell formation. Therefore, NF-*κ*B may serve as a common pathway through which CIH activates multiple atherogenic mechanisms that can synergistically act to cause the onset and development of AS. In addition, elevated plasma levels of several NF-*κ*B target gene products, such as tumor necrosis factor alpha (TNF-*α*), interleukin-6 (IL-6), and vascular cell adhesion molecule-1 (VCAM-1), have been observed in patients with OSAS [71–73]. NF-*κ*B activation not only accelerates the development of metabolic syndrome [74] but also mediates the expression of factor VIII [75] and tissue factor [76], thereby promoting coagulopathies. Thus, NF-*κ*B plays an important role in various AS-promoting mechanisms, such as proinflammatory and procoagulatory processes.

TLR4 is the upstream molecule of NF-*κ*B. As a pattern recognition receptor, it may be involved in the activation of plaque inflammation [77]. Akinnusi et al. [78] demonstrated that TLR4 influenced the activation of the inflammatory response in patients with OSAS. Zeng et al. [79] found that IH could promote TLR4 expression in endothelial cells and TLR4/NF-*κ*B activation, which was followed by the production of inflammatory factors. Furthermore, TLR4 interference not only led to a significant reduction in inflammation but also decreased the AS plaque load and plaque vulnerability by more than half. These findings have helped elucidate the effects of TLR4 on inflammation and atherosclerotic plaque formation, suggesting that IH may promote inflammation by activating the TLR4/NF-*κ*B pathway, thereby inducing AS. Therefore, TLR4 may play an important role in interventions for AS induced by OSAS (or IH) in the near future.

In addition, inflammatory markers such as adhesion molecules and tumor necrosis factor have been strongly associated with atherosclerosis [80, 81]. In clinical studies, Dyugovskaya et al. found that the expression of two adhesion molecules, CD15 and CD11c, was significantly increased in OSA patients compared to controls, and their monocytes adhered more readily to endothelial cells than controls. Treatment with nasal continuous positive airway pressure ventilation significantly suppressed both of these changes [82]. Minoguchi et al. found that TNF-*α* levels were significantly increased in patients with moderate to severe OSAS compared to the other three groups, possibly accelerating the development of atherosclerosis, in a study of healthy people, obese people, patients with mild OSAS, and patients with moderate to severe OSAS. This alteration was independently associated with the duration of hypoxia during sleep. Treatment with nasal continuous positive airway pressure ventilation significantly improved this change [83]. Thus, hypoxia can activate the inflammatory response and promote the development and progression of atherosclerosis through multiple pathways.

### 3.2. Abnormal Platelet Function

Platelet aggregation and activation are abnormally enhanced in patients with OSAS [84, 85]; hence, they play an important role in promoting the pathogenesis of AS and plaque rupture [62]. An increase in OSA severity is associated with an increase in both platelet aggregation and activation [86]. More specifically, IH and reoxygenation can enhance platelet aggregation through substances such as adenosine diphosphate and TNF-*α in vivo* [87, 88]. Furthermore, treatment with continuous positive airway pressure (CPAP) can improve platelet aggregation [84, 89], which may delay the development of AS.

Mean platelet volume (MPV) reflects the average size of circulating platelets and is used to assess platelet activity [90]. It is not only associated with various risk factors for cardiovascular diseases, such as hypertension and diabetes [91], but is also closely related to thromboembolic complications and adverse outcomes of cardiovascular events [92]. MPV has been found to increase with the severity of OSA [93] and was reported to be positively correlated with the apnea–hypopnea index [94, 95]. Meanwhile, patients who underwent uvulopalatal flap surgery showed significantly decreased MPV [96]. Notably, both the frequency and level of nocturnal hypoxemia can promote platelet activation [97], which can have a further impact on AS.

Platelet-derived particles (PMP) are nanoscale fragments released by platelets and are the most abundant particles in human blood, reflecting the degree of platelet activation. Because of its highly procoagulant effect, it has been considered as a prognostic marker for atherosclerosis [98]. Researchers who studied patients with mild OSA versus control subjects without OSA found that patients with mild OSA had significantly higher PMP levels compared to controls [99]. Another study of patients with different degrees of OSAS showed that plasma PMP levels were significantly higher in patients with severe OSAS compared to both patients with mild to moderate OSAS and the normal group, and that PMP levels correlated with AHI. The study also demonstrated that CPAP was able to reduce the level of this particle [100]. All of the above studies can demonstrate the effect of OSA on PMP levels, in which IH plays an important role.

In addition to platelets, coagulation factor levels were also altered in OSA patients. The thrombin-antithrombin (TAT) complex marks the formation of intravascular thrombin, indicating enhanced coagulation. A clinical study showed increased levels of several activated coagulation factors, including TAT, in patients with OSA [101]. As a major coagulation protein, fibrinogen can form insoluble clots or gels when converted to fibrin by thrombin, thus affecting platelet aggregation, and its levels are associated with atherosclerosis [102], which is an important risk factor for cardiovascular disease [103]. Clinical studies have found not only an increase in fibrinogen in patients with OSA, but also a linear relationship between its levels and AHI [104].

### 3.3. Glycolipid Metabolism Disorder

OSAS can alter the patient's metabolic status and significantly increase the incidence of metabolic syndrome [105]; CIH induces abnormal glucose metabolism not only by causing the replication and apoptosis of pancreatic *β*-cells [106, 107] but also by promoting *β*-cell damage and dysfunction [108]. An experimental study [109] found that mice in the CIH group had significantly higher fasting blood glucose and serum insulin levels, compared with mice in the normoxic group, while also exhibiting abnormal glucose metabolism and insulin resistance (IR). The specific mechanisms involved in CIH-mediated IR mainly include reduced phosphorylation, action, and sensitivity of tyrosine kinase (an insulin receptor); inhibition of insulin secretion; and increased production of glucocorticoids and epinephrine [110]. CIH also affects lipid metabolism by increasing the total cholesterol and low-density lipoprotein (LDL) cholesterol (LDL-C) levels in mice, leading to dyslipidemia. Among ApoE^−/−^ mice fed a high-fat diet, those that were also exposed to CIH showed significant differences in AS damage to the aortic sinus and descending aorta compared with normoxic mice [111]. LDL can undergo oxidative modification to produce oxidized LDL (Ox-LDL), which can affect inflammation and AS formation. Studies have demonstrated that the upregulation of Ox-LDL is influenced by CIH [112]. Thus, CIH can mediate the development of AS through an abnormal glycolipid metabolism (see Figure 2).

The current clinical evidence on OSA and dyslipidemia is dominated by cross-sectional studies. Trzepizur et al. found by oxygen saturation index (ODI) in 2081 patients that high triglyceride levels and low HDL cholesterol levels were associated with nocturnal IH and OSA severity and may increase the incidence of cardiovascular disease in patients with OSA [113]. Another clinical study showed that OSA can dynamically increase plasma free fatty acid levels during sleep and that CPAP can attenuate this change, again suggesting an important role for IH in this [114]. This change may be due to the fact that IH regulates hormone-sensitive lipase (HSL) by activating the sympathetic nervous system, thus triggering lipolysis [115].

Recent studies have shown that sex hormones have a regulatory effect on glucose metabolism under CIH conditions. Marcouiller et al. [116] treated mice using either excipients or estradiol and placed them in normoxic or CIH environments, respectively. The results showed that IH impaired glucose tolerance in female mice, particularly in ovariectomized mice, but this effect was reversed by estradiol supplementation, and pancreatic b-cell function was improved. This provides new evidence for improving glycolipid metabolism in the CIH environment.

### 3.4. Oxidative Stress

The continuous and repetitive hypoxia–reoxygenation cycle in CIH causes extensive OS, resulting in endothelial damage and accelerated AS formation [117]. The CIH environment induces the upregulation of peroxidation markers such as malondialdehyde and ROS [118–120]. Of these, excessive ROS can promote VCAM production, leukocyte activation, and systemic inflammation, leading to vascular endothelial damage and dysfunction [110], thereby resulting in the development of AS. In addition, CIH can inhibit endothelial nitric oxide synthase (eNOS) activity and reduce NO levels, causing platelet aggregation and vasoconstriction [121]. Furthermore, metallothionein is a strong antioxidant and is one of the most effective proteins in eliminating free radicals. Under CIH, metallothionein-deficient mice showed more severe arterial inflammation, fibrosis, and oxidative damage, whereas the arterial metallothionein levels of normal mice showed a sharp increase, followed by a decrease. This suggests that CIH mediates OS via the metallothionein pathway [122], thereby promoting the onset and development of AS. In addition, it has been found that the activation of oxidative stress by CIH can be inhibited by progesterone. According to Joseph et al. [123], ovaries of female rats were excised, implanted with osmotic pumps delivering excipients or progesterone, and exposed to room air or CIH, respectively, and divided into three groups: Veh-AIR, Veh-CIH, and Prog-CIH. The results showed that progesterone not only reduced the frequency of CIH-induced apnea and increased hypoxic and hypercapnic ventilatory responses, but also prevented the occurrence of increased NOX activity and decreased cytosolic and mitochondrial SOD activity by CIH. Thus, sex hormones are expected to intervene in the development of related AS by inhibiting CIH-induced oxidative stress.

Cofta et al. responded to oxidative stress levels in OSA patients by plasma total antioxidant status (TAS) and thiobarbituric acid reactive substances (TBARs), which have been shown to be associated with atherosclerosis. This study found that TAS decreased and TBARs increased with increasing severity of OSA [124]. This result is consistent with the findings of Barceló et al. on lipid peroxidation in patients with OSA [125], suggesting the presence of significant oxidative stress alterations in OSA patients.

As one of the intermediate mechanisms of CIH-induced AS, OS also synergistically acts with inflammation, causing damage to the vascular endothelium and hence inducing AS. Tuleta et al. [12] divided ApoE^−/−^ mice into the intermittent air exposure group and the CIH group and found that endothelial function was more severely impaired in the CIH group after 6 weeks; however, they also found that vascular damage can be inhibited by a combination of anti-inflammatory and antioxidant therapy (infliximab + glutathione). Their findings imply that CIH can cause vascular endothelial damage through the synergistic effects of inflammation and OS, which can lead to AS development in severe cases, but it can be effectively treated using combined anti-inflammatory and antioxidant therapy.

### 3.5. Apoptosis

Apoptosis is involved in several pathophysiologic processes and has received increasing research attention as one of the intermediate mechanisms of CIH-induced AS. Apoptosis can suppress injury by attenuating the phagocytosis, migration, and ROS production of neutrophils, whereas delayed apoptosis can exacerbate injury [126–128]. One study [129] reported that IH in patients with OSAS triggered increased neutrophil apoptosis, which induced cardiovascular injury. By conducting *in vitro* experiments on human neutrophils [130], researchers found that IH-treated neutrophils showed an imbalance between Bax of the Bcl-2 protein family (pro-apoptotic) and Mcl-1 (antiapoptotic), as well as prolonged neutrophil survival, which led to persistent inflammation. This process may be affected by the proteolytic enzymes and free radicals released through the interaction of neutrophils and endothelial cells [118]. In addition, lysophosphatidylcholine, one of the components of Ox-LDL, can induce apoptosis in vascular endothelial cells via the p38 mitogen-activated protein kinase (MAPK) pathway, which may lead to AS formation [131].

Survivin is a member of a family of apoptosis inhibitors with complex immunomodulatory effects. A study by Kunos et al. found that plasma survivin was significantly lower in OSA patients compared to non-OSA subjects, correlating not only with OSA severity but also with high BMI, low HDL-C, and high TG levels [132]. This suggests that immune regulation is impaired in OSA patients, and the exact mechanism needs further study and explanation. Klotho is a protein secreted mainly by the kidneys and known for its antiaging properties [133]. Pákó et al. studied plasma klotho levels in OSA patients and non-OSA volunteers and found that CIH decreased the levels of this protein in OSA patients, which may not only promote the development of hypertension but may also have an impact on the inflammatory process [134].

Under IH conditions, the apoptosis of different cells can have different effects on AS. More specifically, insufficient or delayed apoptosis of inflammatory cells can lead to persistent inflammation and contribute to the onset and progression of AS, whereas excessively high levels of apoptosis of vascular endothelial cells can induce IH-mediated cardiovascular diseases. Furthermore, CPAP has been shown to have an ameliorative effect on the apoptosis of vascular endothelial cells [135]. Therefore, apoptosis plays an important role in the process of IH-mediated AS.

### 3.6. Neuroendocrine Disorders

Patients with OSAS experience frequent nocturnal awakenings, IH, and daytime sleepiness, which can lead to sustained excitation of the sympathetic nervous system. This, in turn, increases catecholamine release and activates the renin–angiotensin–aldosterone system (RAAS), resulting in neurohumoral dysregulation. Neuroendocrine abnormalities can accelerate the formation and development of AS in several ways. Trombetta et al. [136] found that patients with multiple sclerosis and OSAS showed stronger muscle sympathetic reflex activation than those without OSAS, which could be attributed to the enhanced peripheral and central chemoreflex responses in OSAS. Other studies [137, 138] have also demonstrated that the occurrence of CIH in patients with OSAS may lead to the inability of the carotid body to maintain a normal dynamic balance of oxygen in the body, which may induce AS through mechanisms involving RAAS upregulation, OS, and inflammatory response in the carotid body.

### 3.7. Small-Molecule RNAs

The occurrence of CIH-mediated AS is accompanied by the abnormal expression of small-molecule RNAs. Most of the existing studies have mainly focused on mRNAs, microRNAs, and long noncoding RNAs. In a study that analyzed the differential expression of mRNAs and long noncoding RNAs in atherosclerotic vascular tissues of ApoE^−/−^ mice, markedly fewer genes were significantly upregulated in mice exposed to CIH for 12 weeks than in mice exposed to CIH for 8 weeks, which leads to weakening of atherosclerotic vascular tissue. The specific mechanism involved was related to the abnormal expression of heat shock proteins caused by CIH via the endoplasmic reticulum protein processing pathway [139]. This study also showed that the long-term CIH exposure resulted in reduced mRNA expression of Rev-erb (a member of the nuclear receptor superfamily that is important for the regulation of immunity, metabolic function, and circadian rhythm) and exacerbated the development of atherosclerosis, suggesting that Rev-erb may be involved in the development of CIH-related AS and play an important role in it. An experiment on male volunteers revealed that after exposure to IH, plasma exosomal microRNAs disrupted the impedance levels while also significantly enhancing the expression of intercellular adhesion molecule-1 and significantly reducing the expression of eNOS in endothelial cells [140]. Thus, IH can alter the exosomes circulating in the body, increase the permeability and affect the function of endothelial cells, and promote the onset and development of AS.

### 3.8. Intestinal Microorganism

There is now growing evidence that gut microbes play an important role in the development of CIH-induced AS. Hu et al. [141] divided ApoE^−/−^ mice into control, AS, and AS+CIH groups and fed them with normal and high-fat diets, respectively. It was found that (i) there was a disturbed gut microbiota in the AS mice; (ii) CIH promoted the development of AS while interfering with the gut microbiota and worsened the disturbed gut microbiota in the mice. Xue et al. [142] used similar experimental methods to confirm the AS-causing effect of CIH and its effect on intestinal microbiota, which may act on the development of AS in various ways, including inflammation and lipid metabolism. Clinical studies have also demonstrated a link between OSA and intestinal flora. Studies in patients with OSA have found altered intestinal epithelial barrier markers and increased intestinal permeability, and this intestinal damage may lead to abnormal lipid metabolism in the liver, which is associated with atherosclerosis [143]. Kheirandish-Gozal, L et al. showed that obese children with OSA had the highest levels of bacterial lipopolysaccharide-binding protein (LBP), a surrogate for intestinal bacterial lipopolysaccharide-induced hypoendotoxemia marker. Therefore, it can be speculated that OSA may disrupt the intestinal microbiota and cause other damage to the body [144].

Therefore, although the mechanisms involved are not yet clear, the link between gut microbes and OSA-associated AS is gradually being recognized and is expected to be used for the prevention and treatment of OSA-associated AS in the near future.

## 4. Advances in Drug Research for OSA-Related AS

New treatment methods are continuously being developed with the gradual increase in the incidence of OSAS. Individuals at a high risk of developing AS require not only correction of IH but also prevention and treatment of AS. Currently, CIH is corrected using nonpharmacologic methods (e.g. CPAP, oral appliances, and sublingual nerve stimulation) supplemented with pharmacologic treatment, whereas the treatment of CIH-related AS is primarily based on drugs, which include drugs for controlling traditional AS risk factors and improving the tolerance of the body to IH. In this section, we will review and summarize the current research advances in the pharmacological treatment of OSA-related atherosclerosis. But most pharmacologic studies related to OSAS are currently in the preclinical stage.

### 4.1. Ethyl Polyenoate

Docosahexaenoic acid (DHA) is an n-3 polyunsaturated fatty acid derived from alternating elongation and desaturation reactions of linolenic acid (a type of essential fatty acid) or eicosapentaenoic acid. This fatty acid is a precursor of several anti-inflammatory lipid mediators (e.g., resolvins and protectins [145]). It has a wide range of actions that can have a role in the regulation of inflammation, thus exerting positive effects [146]. Studies have shown that supplementation with DHA and eicosapentaenoic acid is effective in reducing the production of several pro-inflammatory cytokines, such as IL-6 and TNF-*α*, in healthy individuals [147]. In the study by Van Noolen et al. [148] in ApoE^−/−^ mice, DHA prevented CIH-induced AS. This effect was associated with a decrease in arachidonic acid content in tissues and organs and in aortic matrix metalloproteinase-2 expression caused by the increase in DHA and eicosapentaenoic acid.

### 4.2. *β*3-Adrenoreceptor Agonists

*β*-Adrenoreceptors (*β*ARs) may serve as a new target for the treatment of IH-related AS. Bae et al. [149] found elevated levels of *β*1AR in fetal rat hearts under hypoxic conditions. Arioglu-Inan et al. [150] showed that *β*3AR levels were elevated in patients with cancer, diabetes, and other diseases under hypoxic conditions and also elevated in rat macrophages under IH conditions [151]. As a selective *β*3AR agonist, mirabegron exerts several physiologic effects. It not only relaxes the smooth muscles of the bladder in the treatment of overactive bladder syndrome [152] but also improves left ventricular ejection fraction in patients with heart failure [153–155]. Wang et al. [156] treated ApoE^−/−^ mice with mirabegron and found that mirabegron was able to prevent CIH-induced AS progression. The underlying mechanism was related to the ability of mirabegron to inhibit OS after *β*3AR stimulation.

### 4.3. Statins

Statins are widely used in clinical practice for their lipid-lowering, mainly LDL-lowering, effects. However, in addition to lipid lowering, statins have also been demonstrated to improve endothelial function and to have anti-inflammatory effects [157]. They can inhibit the activation of Rho protein, which increases NOS activity and accelerates its expression, accompanied by an increase in endogenous NO, which ultimately reduces the contraction and proliferation of vascular smooth muscle cells. One study [158] showed that CIH exposure for 14 days in rats led to a wide range of deleterious effects, including blood pressure elevation, OS, and vascular sclerosis, with remodeling of the carotid vessel wall occurring after 28 days, all of which were significantly alleviated by the administration of atorvastatin. Therefore, statins are expected to improve CIH-induced AS.

### 4.4. Propofol

Propofol (2,6-diisopropylphenol) is widely used as an intravenous anesthetic and has been shown to have various anti-inflammatory properties, including inhibition of neutrophil function, alteration of NO production, and reduction of pro-inflammatory cytokine production [159]. Studies have found that the anti-inflammatory effect of propofol is associated with the inhibition of p38 MAPK activation [160]. Li et al. [161] cultured human umbilical vein endothelial cells *in vitro* under an IH/reoxygenation environment, to observe the effects of different propofol doses on NF-*κ*B and HIF-1 activity, as well as on the level of proinflammatory cytokines. Their results showed that 25 and 50 *μ*M propofol had a dose-dependent inhibitory effect on NF-*κ*B activity, which may be based on the inhibition of the p38 MAPK signaling pathway, whereas 100 *μ*M propofol had no significant effect on NF-*κ*B activity. Meanwhile, propofol had no effect on HIF-1 activity regardless of the dose. In addition, 50 or 100 *μ*M propofol had a significant inhibitory effect on various downstream proinflammatory cytokines of NF-*κ*B, such as TNF-*α*, IL-1*β*, and IL-6, under IH/reoxygenation. Thus, propofol may prevent OSAS (CIH)-mediated AS by inhibiting NF-*κ*B-mediated inflammation in vascular endothelial cells.

### 4.5. Chinese Medicine

During the course of research on therapeutic drugs for OSAS or CIH-related AS, marked progress has been made in the field of Chinese medicine. Ma et al. [162] administered a combination of Chinese herbal medicines (ginsenosides and ligustrazine) for supplementing Qi and activating blood circulation to a composite IH- and IR-mediated AS mouse model. Their results showed that ApoE^−/−^ mice in the high-dose group had significantly lower blood glucose, LDL-C, and mRNA and protein expression (TNF-*α*, HIF-1*α*, sterol regulatory element-binding protein 1c [(SREBP-1c], and FAS) levels; significantly higher high-density lipoprotein cholesterol and superoxide dismutase levels; and significantly reduced AS plaque area than mice in the CIH group. This experiment demonstrated that the Chinese herbal medicine combination could significantly improve composite IH- and IR-mediated AS through a number of ways, including regulation of blood lipids and mitigation of inflammation, IR, and OS. The specific mechanism may be related to the inhibition of signaling molecules such as SREBP-1c. This study provides a new basis for the treatment of OSAS (CIH)-related AS with Chinese medicine.

In addition to the drugs mentioned above, salidroside and montelukast have also been shown to have therapeutic effects on CIH-AS (see Table 2).

## 5. Perspective

OSA-CIH generally has adverse consequences in the body, whereas non-OSA-IH exerts different effects under different IH intensities. At present, non-OSA-IH has been applied in sports training to improve exercise tolerance in a hypobaric environment; however, its positive effects remain predominantly reported in animal studies. Future clinical studies conducted in a relatively safe IH environment are warranted to further confirm its positive effects and lay the clinical foundation for its early and widespread application.

With improvements in living conditions, the number of individuals with obesity has steadily increased, and the incidence of OSAS has gradually increased. OSA-CIH can lead to the formation of AS, and IR plays an important role in this process. However, drug research on this pathologic mechanism is scarce, and only a few studies on Chinese medicine are available. Therefore, more studies are needed to fill the gap and provide new evidence for the drug treatment of this disease.

In conclusion, CIH can contribute to the occurrence and development of AS through multiple mechanisms. Since there are no uniform criteria for classifying IH, this paper classifies them into OSA-IH and non-OSA-IH according to whether they are associated with OSA. it is undeniable that there is some irrationality in this classification, but there is no more uniform and reasonable way to classify them. Patients with OSA usually have many coexisting pathologies, such as obesity, diabetes, and hyperlipidemia, and there is no clear evidence that OSA-CIH directly causes AS and further research is needed. The focus of current research is on the indirect aggravation of risk factors by CIH leading to AS, with fewer studies conducted on the direct relationship between CIH and AS. In addition, owing to the complexity of the underlying mechanisms and the interactions among the different mechanisms, it is difficult to clarify the role of a specific mechanism. Furthermore, molecular research on these mechanisms is still in the early stages, involving only a few molecular pathways and insufficient clinical evidence. Therefore, more thorough investigations are needed to gain a better understanding of the pathogenesis of this disease in order to reduce the incidence of complications and mortality.

## Figures and Tables

**Figure 1:** Bidirectional nature of intermittent hypoxia (blue represents the positive effect, red represents the negative effect). The bidirectional nature of intermittent hypoxia means that different patterns of IH can have positive or negative effects on the body. For example, several days of IH training in athletes may improve their tolerance to ischemic hypoxia, whereas patients with OSA or CSA may show multiple pathological outcomes after several months. Animal studies have found that low-frequency, short-duration, mild hypoxia can have a protective effect on the cardiovascular and cerebrovascular system through various mechanisms, while high-frequency, long-duration, severe hypoxia can lead to various pathological outcomes such as abnormal glycolipid metabolism.

**Figure 2:** Possible mechanisms by which OSA-CIH induces atherosclerosis through abnormal glycolipid metabolism (red represents promoted expression and blue represents inhibited expression). OSA-CIH promoted the expression of microRNA-452 in adipose tissue, increased the levels of TNF-*α*, CCL-2, and Resistin; at the same time, it can accelerate lipolysis of white adipose tissue, activation of hypoxia-inducible factor-1, and polarization of macrophages to proinflammatory subtype M1, resulting in the release of more free fatty acids, resulting in fat aggregation; under CIH stimulation, hypoxia-inducible factor-1 (HIF-1) is activated, and lipoangiogenin 4 (Angptl4) is upregulated, leading to the inactivation of lipoprotein lipase (LPL); intracellular mobilization of Ca^2+^ stored in the er and extracellular Ca^2+^ influx play an important role in glucose-induced insulin secretion (GIS). Cyclic ADP-ribose (CADPR) is a second messenger that mobilizes Ca^2+^ from intracellular Ca^2+^ pools. CD38 has the activities of ADP-ribose cyclase and CADPR hydrolase for the synthesis and hydrolysis of CADPR, respectively. In the occurrence of OSA-CIH, CD38mRNA transcription level is significantly inhibited, cADPR level is reduced, and intracellular Ca^2+^ mobilization is impaired, which leads to decreased GIS and may induce T2DM. Studies have shown that OSA-CIH inhibits the expression of glucose transporter 4 (GLUT4) in skeletal muscle, leading to decreased insulin sensitivity and glucose uptake, accelerating the occurrence of T2DM. In addition, OSA-CIH can induce T2DM by promoting the expression of various muscle factors (IL-8, osteonectin, and myonectin). When severe OSA-CIH occurs, liver stearoyl-CoA desaturase 1 (SCD-1) is significantly increased, which increases the secretion of lipoprotein in the body, induces the occurrence of liver lipid peroxidation, and promotes the occurrence of hyperlipidemia. In addition, OSA-CIH also inhibits the expression of microRNA-203 and promotes the expression of selenophenol P to accelerate T2DM.

**Table 1:** Comparison of animal models of OSA-CIH and non-OSA-IH.

Mode of action	OSA-CIH	Non-OSA-IH	
Pneumatic pressure	Atmospheric pressure intermittent hypoxia	Low pressure (exposure to low-pressure, low-oxygen environment for 4-8 hours per day)	Atmospheric pressure intermittent hypoxia
Cycle duration	Short cycle duration (s)	Long cycle duration (h)	Short cycle duration (min)
Inhaled oxygen	Approximately 5–21% FiO_2_	FiO_2_<21%	Approximately 5–21% FiO_2_
Hypoxia duration per cycle	Several seconds	Several hours	Several minutes
Duration of exposure	Several months to several years	Approximately 2–6 weeks	Approximately 2–6 weeks
Effect on the organism	Abnormal liver lipid metabolism [10], liver injury [11],endothelial cell dysfunction [12], hypercholesterolemia, and lipid peroxidation [13]	Positive (low-intensity IH): protects against myocardial ischemia-reperfusion injury [14], prevents arrhythmia [15]	Positive (low-intensity IH): prevents arrhythmia and myocardial infarction [16], improves myocardial contractile function [17], etc.
Clinical features/applications	Seen in patients with OSAS, mostly causes adverse effects	Enhance the physical fitness and training outcomes of athletes [18, 19], relieve coronary heart disease [20]	Improvement/treatment of cognitive dysfunction [21], spinal cord injury [22], chronic obstructive pulmonary disease [23]

Note: Low-intensity IH: 9–16% inhaled oxygen + low number of cycles (3–15 cycles/d) [9].

**Table 2:** Basic research on drugs for the treatment of OSA-related AS.

Drug name	Research subjects	Hypoxic conditions in the experimental group	Intervention period (weeks)	Experimental dose	Mechanism of action
DHA [148]	Male ApoE^−/−^ mice	5–21% FiO_2_, 60 s/cycle, 8 h/d	8	Dietary intake of 0.5% fish oil (containing 80% DHA/4% eicosapentaenoic acid)	AA↓, MMP-2 expression↓ → AS↓
Mirabegron [156]	Male ApoE^−/−^ mice	5–21% FiO_2_, 60 s/cycle, 8 h/d	6	10 mg/kg/d	Nitrotyrosine↓, dihydroglutaraldehyde↓, SOD↑, GSH↑ → OS↓ → AS↓
Atorvastatin [158, 163]	Male C57BL/6 mice	6–21% FiO_2_, 60 s/cycle, 8 h/d	12	5 mg/kg/d	OS↓ → AS↓
	Male Wistar rats	5–21% FiO_2_, 60 s/cycle, 8 h/d	Simultaneous protocol for 2 weeks Delayed protocol for 4 weeks	10 mg/kg/d	
Chinese medicine [162]	Male ApoE^−/−^ mice	(10 ± 0.5%)–(21 ± 0.5%) FiO_2_, 180 s/cycle, 8 h/d	8	Medium dose: 1500 mg Zhenyuan capsule +500 mg ligustrazine phosphate tablet. The high-dose and low-dose groups were administered 2 times and 1/2 of the medium dose, respectively.	LDL-C↓, TNF-*α*↓, HIF-1*α*↓, SREBP-1c↓, FAS↓; SOD↑, HDL-C↑ → blood lipid↓, inflammation↓, OS↓ → AS↓
Montelukast [164]	Male ApoE^−/−^ mice	21–5% FiO_2_, 60 s/cycle, 8 h/d	8	1 mg/kg/d	CysLT 1 receptor blocking → vascular remodeling↓ → AS↓
DMB [165]	Male Ldlr^−/−^ mice; male ApoE^−/−^ mice	21–8% FiO_2_, 0.5–8% CO_2_, 8 min/cycle, 10 h/d	8	1.0%, vol/vol	TMA↓ → TMAO↓ → inflammation, dyslipidemia↓ → AS↓
Propofol [161]	Human endothelial cell line EA.hy926 cells	1% O_2_ 10 min+21% O_2_ 5 min, 15 min/cycle	64 cycles	0, 25, 50, and 100 *μ*M (four concentrations)	p38 MAPK↓ → NF-*κ*B↓, IL-6↓, TNF↓, IL-1*β*↓ → inflammation↓ → AS↓
Salidroside [166]	Male ApoE^−/−^ mice; HUVECs	Hypoxic conditions for mice: 21%–5%–21% FiO_2_, 120 s/cycle, 12 h/d Hypoxic conditions for HUVECs: 21%–5%–21%, 40 min/cycle	7 weeks for mice; 72 cycles for HUVECs	Mice: 100 mg/kg/d; HUVECs: 10 or 100 *μ*M	cAMP/PKA↑ → RhoA/ROCK↓ → ROS↓ → endothelial barrier function↑ → AS↓

GSH: glutathione; SOD: superoxide dismutase; FiO_2_: fraction of inspiration oxygen; AA: arachidonic acid; MMP-2: matrix metalloproteinase 2; DHA: docosahexaenoic acid; SREBP: sterol-regulatory element-binding protein; FAS: a downstream molecule of SREBP-1c; SOD: superoxide dismutase; HDL-C: high-density lipoprotein cholesterol; IHR: intermittent hypoxia/reoxygenation; HUVECs: human umbilical vein endothelial cells; ROS: reactive oxygen species; RhoA: ras homolog gene family member A; ROCK: rho-associated protein kinase; PKA: protein kinase A; CysLT: cysteinyl leukotriene; DMB: 3,3-dimethyl-1-butanol; ApoE^−/−^, apolipoprotein E deficient; Ldlr^−/−^: low-density lipoprotein receptor deficient; IHC: intermittent hypoxia and hypercapnia; RA: room air; HFD: high-fat diet; TMA: trimethylamine; TMAO: trimethylamine N-oxide.

## Data Availability

The data used to support the findings of this study are available from the corresponding author upon request.

## Abbreviations

AS: Atherosclerosis
CIH: Chronic intermittent hypoxia
CPAP: Continuous positive airway pressure
DHA: Docosahexaenoic acid
eNOS: Endothelial nitric oxide synthase
HIF: Hypoxia-inducible factor
IH: Intermittent hypoxia
IL: Interleukin
LDL-C: Low-density lipoprotein cholesterol
MAPK: Mitogen-activated protein kinase
NF-*κ*B: Nuclear factor kappa-B
NO: Nitric oxide
OS: Oxidative stress
OSAS: Obstructive sleep apnea syndrome
Ox-LDL: Oxidized low-density lipoprotein
RAAS: Renin–angiotensin–aldosterone system
ROS: Reactive oxygen species
SREBP-1c: Sterol regulatory element binding protein 1c
TLR4: Toll-like receptor 4
TNF-*α*: Tumor necrosis factor alpha
VCAM: Vascular cell adhesion molecule.
